The article "Identification and Classification of Depressed Mental State for End-User over Social Media" was retracted in 2023. Reasons: signs of a paper mill; suspected computer-generated content; unreliable results or conclusions; lack of ethics approval or compliance.

# Identification and Classification of Depressed Mental State for End-User over Social Media

**DOI:** 10.1155/2022/8755922

**Published:** 2022-04-21

**Authors:** Akhilesh Kumar, Anuradha Thakare, Manisha Bhende, Amit Kumar Sinha, Arnold C. Alguno, Yekula Prasanna Kumar

**Affiliations:** ^1^Department of Information Technology, Gaya College, Gaya, Bihar, India; ^2^Pimpri Chinchwad College of Engineering, Pune, India; ^3^Marathwada Mitra Mandal's Institute of Technology, Pune, India; ^4^Mechanical Engineering Department, Shri Mata Vaishno Devi University Katra, J&K-182320, India; ^5^Department of Physics, Mindanao State University-Iligan Institute of Technology, Tibanga Highway, Iligan City, Philippines; ^6^Department of Mining Engineering, College of Engineering and Technology, Bule Hora University, 144 Oromia Region, Blue Hora, Ethiopia

## Abstract

In researching social network data and depression, it is often necessary to manually label depressed and non-depressed users, which is time-consuming and labor-intensive. The aim of this study is that it explores the relationship between social network data and depression. It can also contribute to detecting and identifying depression. Through collecting and analyzing college students' microblog social data, a preliminary screening algorithm for college students' suspected depression microblogs based on depression keywords, and semantic expansion is researched; a comprehensive lexical grammar was proposed. This research provided has a preliminary screening method based on depression keywords and semantic expansion for college students' suspected depression microblogs, with a screening accuracy. This method forms a depression keyword table by constructing the basic keyword table and the semantic expansion based on the word embedding learning model Word2Vec. Finally, the word table is used to calculate the semantic similarity of the tested microblogs and then identify whether it is a suspected depression microblog. The experimental results on the microblog dataset of college students show that the comprehensive lexical method is better than the SDS questionnaire segmentation method and the expert lexical method in terms of screening accuracy; the comprehensive lexical approach can quickly and automatically screen out a tiny proportion of suspected doubts from a large number of college students' microblogs. Depression Weibo can reduce the workload of experts' annotation, improve annotation efficiency, and provide a suitable data processing basis for the subsequent accurate identification (classification problem) of patients with depression.

## 1. Introduction

Statistics show that there are more than 340 million depression patients in various countries globally and 10 million to 20 million people are suicidal every year [1]. According to the statistics of the Chinese Ministry of Health [2], as of 2012, there were at least 30 million medical records for depression in my country. As a unique group with less social experience, low psychological endurance, and multiple responsibilities for the future family and society, college students have a significantly higher incidence of depression than other groups [3]. The proposed work plays a key role to explore the relationship between social network data and depression. It also contributes to detecting and identifying depression through collecting and analyzing college student's microblog social data.

The article "Identification and Classification of Depressed Mental State for End-User over Social Media" was retracted in 2023. Reasons: signs of a paper mill; suspected computer-generated content; unreliable results or conclusions; lack of ethics approval or compliance.

A survey [4] shows that the penetration rate of Weibo among college students is as high as 90%. Their personality characteristics drive the behavior of users using Weibo, and personality characteristics can be used as one of the clues to infer the psychological characteristics of Weibo users. The Chinese name for “microblog” is “Weibo.” Weibo is a microblogging platform similar to Twitter that is claimed to become the most popular in China. Weibo users express their psychological characteristics such as their views, thoughts, and emotions by publishing online texts. Therefore, the behavior characteristics of users using Weibo and the semantic characteristics of Weibo content may be used to characterize the psychological characteristics of Weibo users. Through in-depth mining and analysis of Weibo users' network texts and logs, the psychological characteristics of users over some time can be obtained, which in turn provides the possibility for analyzing users' mental health status, including depression.

The present article has been planned into various sections. The present section deals with introducing the concept related to depression and its detection.  Section 2 puts light on the discussion of related research work.  Section 3 illustrates the analysis of online social behavior of depression group.  Section 4 describes the preliminary screening algorithm of college students suspected depression microblog based on depression keywords and semantic expansion.  Section 5 describes the Weibo features for depression. The experimental result analysis is described in Section 6, and finally Section 7 portrays the conclusion and possible future works based on the proposed framework.

## 2. Related Work

Psychological analysis with the help of social network data has gradually become a research hotspot. The current research is mainly in two directions. The first research is to explore the relationship between social network data and depression. For example, researchers at the Missouri University of Science and Technology studied the association between Internet usage patterns and depression among college students [5]. The artificial intelligence (AI) can transform medicines and healthcare in profound ways: automation may be used to assess diagnosis patient information, like electrocardiogram, neurology, or x-ray pictures, in order to diagnose illnesses at a preliminary phase based on limited modifications.

The article "Identification and Classification of Depressed Mental State for End-User over Social Media" was retracted in 2023. Reasons: signs of a paper mill; suspected computer-generated content; unreliable results or conclusions; lack of ethics approval or compliance.

The authors in [6] collected data on users with and without depression from Twitter and used the least-squares method to perform regression analysis on the collected data; they counted the time users posted Twitter and analyzed the two types of users. The time difference in posting tweet and the Pearson correlation coefficient method was used to analyze the degree of correlation between user characteristics and depression. The authors in [7, 8] used Facebook data to detect the depression tendency of adolescents. They identified the depressed user through SM rank algorithm, and the source of this data was obtained by collecting and analyzing college student's microblog social data a preliminary screening algorithm for college students' suspected depression microblogs based on depression keywords and semantic expansion.

They analyzed the depression status of college students with the help of psychological diagnostic criteria and Facebook homepage information.

The second research direction is to use social network data to detect and identify depression. For example, the authors in [9, 10] obtained a large amount of Twitter data, used the CES-D scale to get the user's depression state label, and analyzed the user's social network behavior data for feature extraction to construct a depression detection model, proving that Twitter data can be used to detect whether a user has depression. The authors in [11] used data from multiple blog platforms such as Yahoo Japan and Livedoor, combined with Japanese-specific language features for feature extraction. They used machine learning methods to build a depression detection model, proving that blog data can be used to detect depressed users. The authors in [12] found that by analyzing the linguistic content and text structure features of blog texts it is possible to identify the emotional state of network users. The authors in [13] found that it is also possible to identify the emotional state of network users by analyzing the short text content of blogs.

The depression detection and recognition model proposed in the second research belongs to the computer field's classification problem. It is also necessary to manually label the depressed and non-depressed users for training and test set construction. Since manual annotation is time-consuming and labor-intensive, based on the analysis of online social behaviors of depression groups, including network behavior, text semantics (words and topics), etc., this paper proposes a preliminary screening algorithm for suspected depression microblogs.

The article "Identification and Classification of Depressed Mental State for End-User over Social Media" was retracted in 2023. Reasons: signs of a paper mill; suspected computer-generated content; unreliable results or conclusions; lack of ethics approval or compliance.

## 3. Analysis of Online Social Behavior of Depression Group

### 3.1. Data Sources

#### 3.1.1. Weibo Data of Depression Groups

Sina Weibo user “Zuofan,” a depression patient, committed suicide on March 18, 2012, after leaving the last note on Weibo, which had a considerable impact. There are more than one million comments under the last words of this Weibo, and it is still increasing. Therefore, there is no lack of many depressed users in the thread expressing negative emotions. This article obtained the Weibo thread of “Zuofan,” searched for the depression Weibo in the line, and used the Depression Weibo to find depression users. To determine depression microblogs, this paper invited a total of 6 experts engaged in psychology-related work in different industries to mark depression microblogs in the microblogs obtained above independently. In the end, the six experts unanimously identified it as a depression microblog.

Furthermore, a user who publishes more than four depression microblogs at different times is identified as a depression user. Finally, the depression group sample dataset and the depression group Weibo sample dataset are formed [14]. The sample dataset consists of 8,081 depressed users and 90,568 microblogs (including 40,035 depression and 50,533 non-depressed microblogs) published by these users [15]. The obtained microblogs were published in 2014. Until 2018, the acquisition time is January 2019.

#### 3.1.2. Weibo Data of Ordinary College Students

As the college student group concerned in this paper, the microblog data of 53,573 ordinary college students in 8 colleges and universities in the capital were obtained. Considering the research ethics, neither college names nor user names were collected. Instead, a comparative analysis was carried out and used to screen datasets of suspected depression microblogs. This research acquired the “Zuofan” Weibo thread, explored the line for depression Weibo, and utilized the Depression Weibo to locate depression individuals. To identify depression microblogs, this article asked a total of 6 specialists from various sectors who work in psychological to individually mark depression microblogs in the microblogs acquired above. Finally, the six specialists all agreed that it was a depressive microblog [16]. The microblogs were published from November 12, 2018, to December 12, 2018, and acquired in January 2019, with a total of 701,827 microblogs. The microblog data of 8 colleges and universities in the capital are shown in Table 1.

The article "Identification and Classification of Depressed Mental State for End-User over Social Media" was retracted in 2023. Reasons: signs of a paper mill; suspected computer-generated content; unreliable results or conclusions; lack of ethics approval or compliance.

### 3.2. Analysis of Weibo Network Behavior of Depressed Groups

To study how people's post microblogs will change under the influence of depression, this paper uses the microblog sample datasets of the depression group and ordinary college students described in Section 3.1 to compare the depression group and regular college students. It should be noted that the timestamps of 130,210 microblog data of 3 colleges and universities in the ordinary college student group are damaged. The time cannot be accurate to “hours;” this part of the microblog data is discarded, the typical college students used in this section. There are 571,617 group microblog samples.

#### 3.2.1. Analysis of Weibo Posting Behavior of Different Groups

The relationship between the frequency and change rate of Weibo posting and time between the depression group and the general college student group is compared, as shown in Figure 1. The horizontal axis is 24 hours a day, and the frequency of microblog posts on the vertical axis refers to the ratio of the number of seats in a certain period to the total number of seats in the day.

It can be seen from Figure 1 that the general trend of the microblog posting frequency of the depression group and the college student group over time is the same. However, the frequency of posting on Weibo and posting change differs between the depressive group and the general college student group. From 21:00 to about 8:00 the next day, the depression group posted more frequently, and the posting frequency was higher throughout the day. On the one hand, it shows that users with depression are more active than ordinary college students at night and in the early morning. On the other hand, it also shows that users with depression are also their most active periods at night and in the early morning. It can be seen that the activity of the depression group shows a prominent phenomenon of “low day and night high.”

As shown in Figure 1, college students' change rate of postings has apparent fluctuations. Combined with the time distribution of the change rate of postings, the fluctuations occur during getting out of class, lunch, lunch break, and dinner, indicating that the postings of college students are more affected by the actual work and rest. For obvious reasons, the site reflects that the biological clock of ordinary college students is more regulars. On the contrary, the posting change rate of the depression group is relatively flat in the daytime, except for the apparent changes in the early morning and at night, which reflects that the group pays too much attention to themselves, does not want to do things, disregards diet, and even lives passively in life. This phenomenon reflects the characteristics of the depression group accompanied by decreased volitional activity.

The article "Identification and Classification of Depressed Mental State for End-User over Social Media" was retracted in 2023. Reasons: signs of a paper mill; suspected computer-generated content; unreliable results or conclusions; lack of ethics approval or compliance.

### 3.3. Characteristic Analysis of Group Words for Depression

Studies have shown that words with high frequency in documents, namely, high-frequency words, represent the focus of documents to a certain extent. This paper counts and analyzes the high-frequency words and characteristics of Weibo posted by depression groups and ordinary college students and understands the focus of the two types of users. As shown in Table 2, this paper lists the top 20 high-frequency words on Weibo posted by the depression group and the college student group, respectively.

“Language Exploration and Word Techniques” (LIWC) are widely used to study the relationship between word analysis and psychological characteristics. This paper uses the Simplified Chinese version of the “Language Exploration and Word Technology” (SC-LIWC) tool [17] to analyze the word characteristics of the depression group as follows:

- Depressed groups use the first-person singular pronoun “self” most frequently in Weibo texts. The above phenomenon shows that the self-awareness or self-perception of the depressive group is too firm, and they are more immersed in their world in social life and are reluctant to connect with other people.
- Depressed groups use the exact word “really” with a high frequency in Weibo texts. This shows that patients with depression are more likely to go to extremes in their views of the world and are more likely to see the world in a “black or white” concept.
- Depressed groups also use negative words “no,” “do not want,” and “but” in Weibo texts more frequently. This phenomenon shows that this group often has negative emotions in social life, and then they are more likely to deny themselves, view the world negatively, and treat life negatively.
- In addition, depressive groups also widely use function words and filler words with no actual meaning in Weibo texts. This phenomenon shows that the group has the problem of imprecise and unclear thinking, and then it reflects the psychological characteristics of the group such as hesitation and contradiction.

In contrast, the words frequently used by ordinary college students in Weibo texts are mostly social process words (“reply,” “repost”), positive emotion words (“hahaha,” “like”), and proper nouns (“Weibo” “Zhu Yilong,” “Chaohua,” “Bu Fan,” “You Changjing,”, “Mickey”), and so on. This shows that ordinary college students are more concerned about the outside world and social hotspots, and they are more connected with the outside world and interact with others in social life. These characteristics reflect the group's upbeat, optimistic, and other psychological factors.

The article "Identification and Classification of Depressed Mental State for End-User over Social Media" was retracted in 2023. Reasons: signs of a paper mill; suspected computer-generated content; unreliable results or conclusions; lack of ethics approval or compliance.

### 3.4. Topic Analysis of Depression Groups

Studies have shown that the text's topic content reflects the text's central idea to a certain extent [18]. Therefore, this paper will extract the topic content of Weibo posted by depression groups and analyze its implicit main idea. We use Linear Discriminant Analysis (LDA) [18] to model the topic of the depression group and the number of issues is set to 20. The Latent Dirichlet Allocation (LDA) method is an autonomous learning method that tries to classify a set of measurements into a number of separate groups. The most frequent use of LDA is to find a user-specified number of topics from those articles that are in a textual collection. It is also a creative statistic framework that enables unidentified entities to describe why certain sections of the dataset are similar. The results showed that most topics reflected the four aspects of the psycho-emotional disorder, somatic disorder, psychomotor disorder, and psychological disorder in patients with depression. The above content is highly consistent with the four dimensions of depression assessment questionnaires such as SDS. This paper selects five topics for analysis, as follows. The five topics and key words of selected depression groups are shown in Table 2.

- Topic 1. Lonely topic: depressed patients are lonely and feel that they have no one to talk to. A psycho-affective disorder can be classified as depression.
- Topic 2. Choose a topic of death anxiety. This may be related to patients with severe depression whom the disease has tortured for a long time, hoping to be relieved but afraid of death, so they prefer to end their lives suddenly in an accident. This is a typical psychological symptom of patients with severe depression, classified as a psychological disorder of depression.
- Topic 3. I hate my topic. Feeling that oneself is a waste, garbage, useless, and dispensable are typical symptoms of patients with depression, which can be classified as psychomotor disorders.
- Topic 4. The topic of sleep disorders. Insomnia is a specific symptom of depression and can be classified as a somatic disorder of depression.
- Topic 5. A topic that encourages you to persevere. This may be related to the positive side of depression patients in the process of fighting depression and receiving treatment, cheering, and promoting themselves. In addition to topic 5, some cases also reflect positive issues such as depression treatment and social support for depressed patients. However, these topics are not reflected in the evaluation questionnaire. Therefore, it can be regarded as a microblog text different from traditional depression, such as questionnaire evaluation—the difference in detection.

The article "Identification and Classification of Depressed Mental State for End-User over Social Media" was retracted in 2023. Reasons: signs of a paper mill; suspected computer-generated content; unreliable results or conclusions; lack of ethics approval or compliance.

## 4. Preliminary Screening Algorithm of College Students' Suspected Depression Microblog Based on Depression Keywords and Semantic Expansion

This algorithm first establishes the basic keyword table of depression and then uses the Word2Vec tool to expand the vocabulary further to obtain the extended keyword table for depression. The flow of the algorithm is shown in Figure 1. To find the best algorithm, this study used three different methods to establish the depression basic keyword table and the corresponding depression extended keyword table for comparison. The current method plays a crucial role to explore the link between social network data and depression. The proposed research is more accurate than existing approaches like the SDS questionnaire segmentation method and the expert lexical method in terms of accuracy. The comprehensive lexical approach can quickly and automatically screen out a tiny proportion of suspected doubts from a large number of college students' microblogs.

### 4.1. Generation of Essential Keywords for Depression

  Method 1. SDS questionnaire segmentation method refers to using the “jieba” text segmentation tool to segment the Depression Self-Rating Scale (SDS) and the segmentation result as the primary keyword table for depression. First, half of the items representing positive emotions in the SDS scale were converted into objects representing negative emotions. Next, all things were divided into words. Words such as subject and modal particles were removed to obtain a vocabulary consisting of 47 words (such as feeling, mood, depression, depression, morning, mood, crying, etc.).
  Method 2. The expert vocabulary refers to brainstorming strategies by several experts to conduct brainstorming based on the four dimensions of psycho-emotional disorders, physical disorders, psychomotor disorders, and psycho-behavioral disorders by using research experience and obtaining a primary keyword list for depression. It consists of 238 words (e.g., low mood, depression, depression, and sullenness, insomnia, waking up quickly, nightmares, loneliness, heavy day and night, etc.).
  Method 3. Synthetic lexicon, the depression essential keyword list of the synthetic glossary, is the same as the expert lexicon. Then the essential dictionary is expanded according to the method in Section 3.2 to form the depression expanded keyword list.

The article "Identification and Classification of Depressed Mental State for End-User over Social Media" was retracted in 2023. Reasons: signs of a paper mill; suspected computer-generated content; unreliable results or conclusions; lack of ethics approval or compliance.

### 4.2. Generation of Word2Vec Semantic Expansion and Depression Expansion Keyword Table

The method of Word2Vec semantic expansion is as follows: calculate the cosine similarity between each word of the depression basic keyword table in the previous step and all the words in the dictionary, and take the top 10 words with the most significant similarity as the synonym of the word. In this way, each word in the primary keyword table can be screened for ten words close to it, duplicated, and then words unrelated to depression or words that do not meet the experimental requirements, such as English words and codes, are manually removed. Depression Extended Keyword List: the Python synonyms package was called during the experiment, and synonyms used the word vectors trained by Wiki data-corpus to generate a synonym table.

It should be noted that the expanded keyword list of depression obtained by comprehensive lexical grammar is a word list generated by adding drug names related to depression based on expanded keywords of depression in expert lexical grammar. This study lists the chemical names and trade names of all drugs currently on the market to treat depression, such as agomelatine, amoxapine, Bristol-Myers Squibb, Prozac, phenelzine, Malak, imipramine, trazodone, etc. 74 kinds. After expanding the three essential word lists, 392, 474, and 548 keyword lists for depression were obtained.

### 4.3. Similarity Analysis

Taking the microblog data of ordinary college students in Section 2 as a sample, screening for depression first, we need to perform preprocessing on Weibo, such as deleting modal words, word segmentation, etc., and then perform similarity analysis. The similarity calculation method divides each microblog into *A*_1_, *A*_2_, *A*_*m*_, and each word segment. The word vector *K*_1_, *K*_2_, *K*_*m*_ of the concave extended keyword table calculates the cosine similarity one by one. The cosine similarity value is used to correlate word segmentation and depression. For example, in the microblog word segmentation *A*_1_, the cosine similarity between *A*_1_ and *K*_1_, *K*_2_,…, *K*_*n*_ and other *n*-words is obtained in turn, and the largest one of the *n* cosine similarities is taken as the correlation between the word and depression. The screening criteria for suspected depression microblogs are as follows: take the average of the top 3 microblogs with the highest similarity between microblogs *A*_1_, *A*_2_,…, *A*_*m*_ and the depression keyword table (after many manual tests, 3 are better). If the average value is higher than 95%, Weibo is considered to be related to depression. If the number of word segments in Weibo is less than 3, calculate the average of all words.

The article "Identification and Classification of Depressed Mental State for End-User over Social Media" was retracted in 2023. Reasons: signs of a paper mill; suspected computer-generated content; unreliable results or conclusions; lack of ethics approval or compliance.

## 5. Weibo Features for Depression

Since the behavior of Weibo users is mainly affected by two factors, their cognitive level and network environment, the influence of users in this paper consists of two aspects: the initial value of the user's power and the influence of the user's behavior at different times. The initial value of the user's mark is mainly calculated by the number of users' followers and the number of microblogs posted by the user before the topic spreads. The behavioral impact of the user at time *t* is calculated through the user interaction network at time *t*. The user interaction network at time *t* is divided into users at time *t*.

Existing research on microblog communication usually uses users as nodes and attention among users and fans as edges to build a user relationship network. However, reducing the impact of redundant node information (such as zombie nodes) on research does not directly rely on attention. Instead, we build a network with fan information but rely on users' forwarding, comments, and likes in different moments of Weibo topics to build a network. To facilitate the description of the problem, here are the following definitions.

**Definition 1 .**

(user forwarding relationship network at time *t* in microblog topic). The user forwarding relationship network is represented by a two-tuple *H*_1*t*_ = (*V*_1*t*_, *F*_1*t*_, *X*_1*t*_) where *H*_1*t*_ represents the user forwarding relationship network at time *t* in the microblog topic, *V*_1*t*_ represents all users participating in the case at time *t*, *F*_1*t*_ represents the edge set in the network, and each edge in the edge set represents the existence of the existence between two users.

Forwarding relationship, *X*_1*t*_ is the forwarding weight of the directed edge.

**Definition 2 .**

(the network of user comments and likes in the microblog topic at time *t*). The network of user comments and likes is represented by a two-tuple *H*_2*t*_ = (*V*_2*t*_, *F*_2*t*_, *X*_2*t*_) where *H*_2*t*_ represents the user comments of the microblog topic at time *t*, *V*_2*t*_ represents all users participating in the case at time *t*, *F*_2*t*_ represents the edge set in the network, each edge in the edge set represents a comment, or like of the relationship between two users, *X*_2*t*_ is the comment of the directed edge like weight.

**Definition 3 .**

(user influence). The user influence in the microblog topic is represented by a quadruple *J* = (*H*, *V*, *J*_*t*_, *f*), where *H* includes *H*_1*t*_ and *H*_2*t*_, U represents the set of users participating in the topic, which indicates the user's influence at time *t*, and *f* is the mapping relationship of each element in the quintuple I. The definition of the influence of the user *w*_*i*_ is as follows:

(1) $$\begin{array}{c} J\left(w_{i}\right)=f\left(J_{t}\left(w_{i}\right)\right),\;w_{i}\in V. \end{array}$$

The article "Identification and Classification of Depressed Mental State for End-User over Social Media" was retracted in 2023. Reasons: signs of a paper mill; suspected computer-generated content; unreliable results or conclusions; lack of ethics approval or compliance.

### 5.1. Swarm Model Definition

In the Swarm model, the agent interacts with other individuals entirely according to its judgment in the environment where the group has no control centre, thereby influencing the whole. Like the agent in the Swarm model, any user in the microblog topic can participate in the functions of posting microblogs, following interactions, commenting, and liking and the interaction between users will also affect the behavior of individuals. According to the similarity between user interaction in Weibo topic and agent communication in Swarm model, the Swarm model is integrated into the Weibo topic user influence evaluation algorithm. The key is to flexibly combine users to publish Weibo, forward, and comment in agent movement and compliments.

Based on the calculation method proposed by Specter and Klein in the literature [12], according to the research content of this paper, the physics of the Swarm model is redefined here.

Meaning, before giving definitions, first understand the following two concepts.

In the microblog topic, the *w*_*i*_ user's neighborhood user node at time *t* refers to the user set that has a more significant impact on the user *w*_*i*_. It is the set of users who forward the user *w*_*i*_ microblog. The neighborhood users of the user *w*_*i*_ are different at different times. It can be obtained from the statistics of the user forwarding relationship network at the moment *t* of the microblog topic.

User nodes around the *w*_*i*_ user at time *t* in the microblog topic refer to the set of users that impacts the user *w*_*i*_, but the impact is not very large. It is a set of users who comment and like the user *w*_*i*_ Weibo. At different times, the users around the user ui are other and based on the microblog topic. The user at time *t* is statistically derived from the network of comments and likes.

**Definition 4 .**

(Swarm model for Weibo topics)

(1) In the Swarm model, *Y*_1_ represents the mean vector of an agent pointing to all agents far away from its ranged. In Weibo, the neighborhood user nodes of the user *w*_*i*_ are used for calculation, and the analysis is carried out through the user forwarding relational network, calculated as follows:
  (2) $$\begin{array}{c} Y_{1t}=\sum_{y\in V}J_{t-1}\left(y\right)*\left(X_{1t}\left(yw_{i}\right)\right),\\ X_{1t}\left(yw_{i}\right)=\frac{Q_{t}\left(yw_{i}\right)}{U\left(yw_{i}\right)}. \end{array}$$
Among them, *V* is the set of users participating in the microblog topic, *J*_*t*−1_ (*y*) is the user influence of user *y* at the last moment, (*X*_1*t*_(*yw*_*i*_)) is the contribution *t* of user *y* to user *w*_*i*_ Weibo forwarding, *Q*_*t*_(*yw*_*i*_) is the number of microblogs forwarded by user *y* to user *w*_*i*_ at time *t*, and *U*(*yw*_*i*_) is the total number of microblogs delivered by user *v* to all users in the topic at time *t*.
(2) *Y*_2_ is the vector in the Swarm model that points to the centre of the simulated world and is represented by the average of the top 20% of user influence in the last iteration of Weibo user influence evaluation. The calculation is as follows:
  (3) $$\begin{array}{c} Y_{2t}=\;\frac{\sum_{y\in \text{Top}}J_{t-1}\left(y\right)}{n}. \end{array}$$
Among them, Top is the top 20% user set at the last moment, and *n* is the number of Top users.
(3) *Y*_3_ is the average velocity vector of all agents around a particular agent. It is expressed by the moderate influence of user nodes around the user *w*_*i*_ on the user. The calculation formula is as follows:
  (4) $$\begin{array}{c} Y_{3t}=\;\sum_{y\in V}J_{t-1}\left(y\right)*\;\left(X_{2t}\left(yw_{i}\right)\right)\;,\\ X_{2t}\left(yw_{i}\right)=\;\frac{C_{t}\left(yw_{i}\right)}{U_{2t}\left(yw_{i}\right)}. \end{array}$$
Among them, *X*_2*t*_(*yw*_*i*_) is the contribution of user *y* microblog comments and likes to user *w*_*i*_ at time *t*, *C*_*t*_(*yw*_*i*_) is the number of comments and likes of user *y* to user *w*_*i*_ at time *t*, and *U*_2*t*_(*yw*_*i*_) represents the total number of comments and likes of user *y* at time *t*.
(4) *Y*_4_ is the vector that an agent points to the centre formed by all the agents around it. The calculation formula given in this paper is as follows:
  (5) $$\begin{array}{c} Y_{4t}=\;\frac{\sum_{y\in V}J_{t-1}\left(y\right)}{N}. \end{array}$$
Among them, *N* is the number of all users in the topic.
(5) *Y*_5_ is a random unit-length vector, which is not considered in calculating Weibo user behavior influence.

The influence formula of user *w*_*i*_ at time *t* is expressed as

(6) $$\begin{array}{c} J_{t}w_{i}=b1*Y_{1t}+\;b2*Y_{2t}+\;b3*Y_{3t}+b4*Y_{4t}. \end{array}$$

The article "Identification and Classification of Depressed Mental State for End-User over Social Media" was retracted in 2023. Reasons: signs of a paper mill; suspected computer-generated content; unreliable results or conclusions; lack of ethics approval or compliance.

## 6. Experimental Result Analysis

### 6.1. Screening Effectiveness Analysis

Since the expert lexicon and the comprehensive lexical method are only proper nouns without drugs, there is no need to compare the three algorithms in pairs to determine the optimal way. Instead, the performance on the blog can be reached and then compared with the microblogs screened out by the comprehensive lexical medicine proper nouns compared with the expert lexical ones. The comprehensive lexical method is different from existing methods in term of accuracy; the proposed method can quickly and automatically screen out a tiny portion of suspected doubts from large number of college students microblogs. This paper randomly selects 2% of the microblog screening results of the two algorithms of the SDS questionnaire segmentation method and comprehensive verbal method and submits it to experts to determine whether the screening results are valid.  Table 3 shows the expert evaluation results of the linguistic segmentation method and comprehensive lexical method of the SDS questionnaire.

The following five microblogs are all screened in the whole language rather than expert speeches based on comparing vocabulary and specialist vocabulary.

- Is there any food that can clear away heat, reduce fire, and detoxify? Huang Lianpo has been too irritable recently.
- Facts have proved that depression does not equal unhappiness.
- Harvard Brain Scientist: if you are not good at studying and feel depressed, a more effective way than taking medicine is…
- I am also recently often depressed and uncontrollable.
- Fentanyl that became popular overnight, the black swan has come again, are Renfu Pharmaceuticals and Renhua Pharmaceuticals at risk? On Sunday morning, fentanyl was unexpectedly the most critical market focus for December. Suppose previous protests against fentanyl in the US and Canada failed to attract domestic investors' attention. In that case, the fentanyl released today will undoubtedly be prevalent again and again. From the perspective of the North American market, the ferocity and danger of fentanyl have been elevated to the “opium” war.

It can be seen from the above five items that the comprehensive lexical method adds a certain amount of noise to the expert verb form (such as items (1) and (5), items (2), (3), and (4)) with negative emotion.

To sum up, comparing the three algorithms, the comprehensive vocabulary method performed the best in screening suspected depression microblogs. Compared with the expert lexicon, although a certain amount of noise will be introduced after introducing the drug name dimension, which increases the misrecognition rate, it is possible to screen out suspected depression microblogs missed by the expert lexicon. Furthermore, after expanding the scope of the sample set, we can directly screen out the relevant microblogs that meet the depression treatment drugs in the microblogs.

### 6.2. Comparison of Impact Coverage

The user depression coverage of top *k* is compared, and the experimental results are shown in Figure 2 with Table 4. The results show that the SM rank algorithm can effectively find users with high depression rank in Weibo topics. The impact coverage rate of depression analysis is shown in Table 4.

The article "Identification and Classification of Depressed Mental State for End-User over Social Media" was retracted in 2023. Reasons: signs of a paper mill; suspected computer-generated content; unreliable results or conclusions; lack of ethics approval or compliance.

### 6.3. Depression Comparison in Different Periods

This paper proposes that the SM rank algorithm can calculate the depression of different users in different periods, where the period is set to days. The period can be set to a shorter or longer time (such as two *h*, six *h*) according to different datasets in one month; Figures 3 and 4 show the daily depression curves of the top 5 users on other datasets, respectively. It can be seen that the depression of each user is distinct at different times; the daily depression of the top five users in gene editing is shown in Figure 3, where user 1 and user 4 have a significant depression on the first day, but their impact decreases in the next two days, indicating that the user is the topic of the microblog. The initiators of user 2, user 3, and user 5 had more depression on the second day, and they were the leading communicators of the topic. The daily depressions of the top five users in food safety are shown in Figure 4, where user 2, user 1, user 4, and user 5 had a more significant depression on the first day, indicating that they played an essential role in initiating Weibo topics. In contrast, user 1 and user 3 depression level *d* is in the middle. If it is larger, it means that they are the primary communicators of this Weibo topic; on the last day, when the popularity of the event decreases and is about to die, the depression of all users decreases. The above conclusion is similar to the situation in the entire network.

## 7. Conclusion

The depression group sample dataset and the depression group microblog sample dataset were constructed, and the microblog data of ordinary college students were collected. Based on this, we analyzed and summarized the characteristics of social network behaviors such as network behavior and text semantics (words and topics) of depression groups publishing Weibo. Based on these characteristics, expert wisdom was synthesized. This research is very useful to explore the relationship between social network data and depression. It also detected and identified depression through collecting and analyzing college students' microblog social data. The Word2Vec tool was used to establish an extended keyword list for depression, which supported the study to propose a preliminary screening algorithm for microblogs suspected of depression. The experimental outcoming on the microblog dataset of college students shows that the comprehensive lexical method is better than the SDS questionnaire segmentation method in terms of screening accuracy, and the screening accuracy rate is 65.7%. This paper presents a preliminary screening algorithm for college students' suspected depression microblogs, based on depression keywords and semantic expansion. Although the accuracy rate is not very high, it can quickly screen microblogs with depressive emotions from many college students' microblogs, reduce the workload of experts' labeling, improve the labeling efficiency, and further accurately identify subsequent depression patients (classification problem) to provide a sound basis for data processing. To improve the screening accuracy, the first recognition error and the second recognition error were analyzed and discussed, respectively. Optimizing the algorithm combined with semantic context analysis will be proposed in the future [19].

The article "Identification and Classification of Depressed Mental State for End-User over Social Media" was retracted in 2023. Reasons: signs of a paper mill; suspected computer-generated content; unreliable results or conclusions; lack of ethics approval or compliance.

## Figures and Tables

**Figure 1:** Identify algorithm steps.

**Figure 2:** Impact coverage rates of depression analysis.

**Figure 3:** Daily depressions of the top 5 users in “gene editing.”

**Figure 4:** Daily depressions of the top 5 users in “food safety.”

**Table 1:** Microblog data of 8 colleges and universities in the capital.

School	Number of posts	User number
1	117 844	9858
2	231 004	16855
3	64822	5656
4	61802	5418
5	120281	5506
6	56987	627
7	13484	2618
8	19893	7302

**Table 2:** 5 topics and key words of selected depression groups.

Topic ID	Topic heading
Topic 1	No friends, lonely, no one to chat, need a place to go out, there are people around
Topic 2	Fear of death, despair, relief, accident, face the terrible future, dare not now
Topic 3	You and others are disgusting, useless, garbage, you only want to disgust
Topic 4	Today I cannot sleep till tomorrow, I cannot eat at night
Topic 5	Live hard, hope, come on, persist in pain, continue to live, see, live

**Table 3:** Expert evaluation results of screening algorithm.

Evaluation item	SDS questionnaire segmentation method	Synthetic lexical
The total number of Weibo identified as suspected depression	90771	20731
Randomly select 2% of the number of Weibo	1900	415
Experts determine the number of Weibo with obvious negative emotions	98	275
Proportion (%)	5.088	68.70

**Table 4:** Impact coverage rates of depression analysis.

Serial number	SMS rank	Page rank	Fans rank	Repost rank
1	0.2	0	0.1	0.1
2	0.2566	0.003	0.1349	0.1562
3	0.31	0.0268	0.1457	0.1789
4	0.3698	0.0298	0.1562	0.2145
5	0.3897	0.0311	0.1889	0.2598
6	0.4059	0.0388	0.2245	0.2897
7	0.4256	0.065	0.2598	0.3157
8	0.4455	0.0989	0.2997	0.3489
9	0.4892	0.1115	0.3257	0.3645
10	0.51	0.1256	0.3489	0.3985
11	0.5213	0.2596	0.3545	0.4258
12	0.5805	0.2999	0.3985	0.4356
13	0.6156	0.3986	0.435	0.4459
14	0.6325	0.4515	0.4356	0.5126
15	0.6589	0.4698	0.4459	0.5569
16	0.6685	0.4817	0.5126	0.6599
17	0.6899	0.4978	0.5526	0.6899

The article "Identification and Classification of Depressed Mental State for End-User over Social Media" was retracted in 2023. Reasons: signs of a paper mill; suspected computer-generated content; unreliable results or conclusions; lack of ethics approval or compliance.

## Data Availability

The data shall be made available on request.
